The article "Hsp90β is involved in the development of high salt-diet-induced nephropathy via interaction with various signalling proteins" was retracted in 2021. Reasons: manipulated images; duplicated images; original data or images not available.

# Hsp90β is involved in the development of high salt-diet-induced nephropathy via interaction with various signalling proteins

**DOI:** 10.1098/rsob.150159

**Published:** 2016-04-20

**Authors:** Shi-hai Yan, Ning-wei Zhao, Wei-min Jiang, Xin-tong Wang, Si-qi Zhang, Xuan-xuan Zhu, Chun-bing Zhang, Yan-hong Gao, Feng Gao, Fu-ming Liu, Zhu-yuan Fang

**Affiliations:** 1 Affiliated Hospital ofNanjing University of Chinese Medicine, Jiangsu Province Hospital of TCM, Nanjing, People's Republic of China; 2 Shimadzu Biomedical Research Laboratory, Shanghai, People's Republic of China; 3 Nanjing Normal University, Nanjing, People's Republic of China

**Keywords:** high salt-diet-induced nephropathy, WKY, SHR, Hsp90β

## Abstract

A high-salt diet often leads to a local intrarenal increase in renal hypoxia and oxidative stress, which are responsible for an excess production of pathogenic substances. Here, Wistar Kyoto/spontaneous hypertensive (WKY/SHR) rats fed a high-salt diet developed severe proteinuria, resulting from pronounced renal inflammation, fibrosis and tubular epithelial cell apoptosis. All these were mainly non-pressure-related effects. Hsp90β, TGF-β, HIF-1α, TNF-α, IL-6 and MCP-1 were shown to be highly expressed in response to salt loading. Next, we found that Hsp90β might play the key role in non-pressure-related effects of salt loading through a series of cellular signalling events, including the NF-κB, p38 activation and Bcl-2 inactivation. Hsp90β was previously proven to regulate the upstream mediators in multiple cellular signalling cascades through stabilizing and maintaining their activities. In our study, 17-dimethylaminoethylamino-17-demethoxygeldanamycin (17-DMAG) or Hsp90β knockdown dramatically alleviated the high-salt-diet-induced proteinuria and renal damage without altering blood pressure significantly, when it reversed activations of NF-κB, mTOR and p38 signalling cascades. Meanwhile, Co-IP results demonstrated that Hsp90β could interact with and stabilize TAK1, AMPKα, IKKα/β, HIF-1α and Raptor, whereas Hsp90β inhibition disrupted this process. In addition, Hsp90β inhibition-mediated renal improvements also accompanied the reduction of renal oxidative stress. In conclusion, salt loading indeed exhibited non-pressure-related impacts on proteinuria and renal dysfunction in WKY/SHR rats. Hsp90β inhibition caused the destabilization of upstream mediators in various pathogenic signalling events, thereby effectively ameliorating this nephropathy owing to renal hypoxia and oxidative stress.

## 1. Introduction

A long-time phenomenon has been observed and confirmed that hypertensive patients from northern China usually suffer from more serious kidney disease than those from southern China, mainly because people in northern China favour a high-salt diet, whereas people in southern China do not.

The article "Hsp90β is involved in the development of high salt-diet-induced nephropathy via interaction with various signalling proteins" was retracted in 2021. Reasons: manipulated images; duplicated images; original data or images not available.

Based on previous investigations, high-salt diet often increases glomerular filtration rate, proteinuria, size and weight of rat kidneys [1]. However, it was found that the augmented proteinuria was not simply owing to the adverse effects of hypertension on kidneys. Atenolol treatment was reported to reduce systolic blood pressure (SBP) effectively, but it hardly relieved the increased urinary protein excretion in salt-loaded SHR, suggesting blood-pressure-independent factors possibly contribute to renal disease. Thus, it was concluded that the increases in SBP and proteinuria might be independent consequences of a high-salt diet [2]. In addition to the well-known effect of salt loading on blood pressure, such clinical and experimental observations were in favour of non-pressure-related effects of salt that could contribute to its influence on nephropathic outcome [3].

A reduction in renal oxygenation often occurs in most chronic kidney diseases irrespective of aetiology. This is due to a combination of several pathophysiological and morphological changes, which consist of increased oxygen demand from hyperfiltration, tubular hypertrophy, capillary rarefaction and glomerular injury. The resulting reduction in renal oxygen availability is furthermore exacerbated by renal fibrosis, which limits oxygen diffusion [4,5]. Hypoxia-inducible factor-1α (HIF-1α) is a hallmark of tissue hypoxia, which is responsible for the induction of genes that facilitate tissue fibrosis from normoxia to hypoxia [6]. Among numerous growth factors and cytokines, transforming growth factor-β (TGF-β) has been identified as the most potent target cytokine of HIF-1α in renal fibrosis [7,8].

On the other hand, HIF-1α levels paralleled not only tissue hypoxia, but also oxidative stress and accumulation of inflammatory mediators, such as tumour necrosis factor-α (TNF-α), interleukin-6 (IL-6) and monocyte chemotactic protein 1 (MCP-1) [9]. IL-6^−/−^ mice previously demonstrated reduced histological evidence of tubular injury when they were subjected to renal infusion/repression (I/R) [10]. In the kidney, TNF-α often contributes to the chronic inflammation that often precedes interstitial matrix deposition, and is also implicated in obstruction-induced renal tubular cell apoptosis [11]. MCP-1 has been recognized as an angiogenic cytokine, which was implicated in the pathogenesis of multiple diseases characterized by monocytic infiltrates, such as psoriasis, rheumatoid arthritis or atherosclerosis. Furthermore, MCP-1 was likewise produced in renal tubular cells, and increased MCP-1 expression usually contributed to renal tubular damage [12].

The article "Hsp90β is involved in the development of high salt-diet-induced nephropathy via interaction with various signalling proteins" was retracted in 2021. Reasons: manipulated images; duplicated images; original data or images not available.

Although hypoxia is well known to increase HIF-1α, a growing body of evidence indicates that oxidative stress-dependent mediators, including inflammatory cytokines and growth factors, also stimulate HIF-1α gene activity [13]. In short, high-salt-induced nephropathy is an extremely complicated biological process, which contains the cross-talk between renal hypoxia and excessive oxidative stress. Thus, animal models were much better research objects than cell models in this study.

Urine is easily obtainable biological fluid that contains useful biological markers for renal diseases. It has been widely used to study renal pathophysiology. Urinary proteins mainly come from the glomerular filtration of blood plasma. Urine has been defined as a fluid biopsy of the kidneys because it provides direct (and indeed substantial) information about the kidney. Thus, many changes and alterations in kidney functions can be detected in the urinary proteome [14]. Here, with the help of the latest proteomic technology, we investigate the possible mechanisms of high-salt-diet-induced nephropathy in normotensive Wistar Kyoto (WKY)/spontaneous hypertensive (SHR) rats.

## 2. Material and methods

### 2.1. Antibodies and reagents

Primary antibodies against Hsp90β, TAK1, p-TAK1 (phospho-T187), TAB-1, ERK1/2, p-ERK1/2 (ERK1: phospho-Y204, ERK2: phospho-Y187), JNK1/2, p-JNK1/2 (phospho-T183/Y185), p38, p-p38 (phospho-T180/Y182), IκBα, p-IκBα (phospho-S32/S36), NF-κB p65, Bcl-2, cytochrome *c*, p-Bcl-2 (phospho-S87), p-p70S6 K (phospho-T389), p-mTOR (phospho-S2448), IKKα/β, p-IKKα/β (phsopho-S176/S177), HIF-1α, Lamin B1 (internal standard in nuclear protein fractions), β-actin (internal standard in cytosolic protein fractions) were from Abcam. Monoclonal antibodies against MKK3/6, p-MKK3/6 (MKK3: phospho-S189, MKK6: phospho-S207), AMPKα and phospho-AMPKα (phosphor-T172) were from Cell Signaling Technology and R&D Systems, respectively. Control rabbit IgG was from Santa Cruz Biotechnology. Horseradish peroxidase-conjugated secondary antibodies were obtained from Calbiochem. Secondary antibodies coupled to IRDye800 fluorophore for use with the Odyssey Infrared Imaging System were purchased from Rockland. Hsp90 inhibitor, the water-soluble 17-DMAG, was purchased from Sigma Aldrich.

### 2.2. Animal protocols

All rats purchased from Charles River (Wilmington, MA) were maintained in animal facilities of Jiangsu Province Hospital of Chinese Medicine and allowed free access to rodent feed and tap water. At first, eight-week-old male SHR rats (*n* = 40) and WKY rats (*n* = 40) were used. SHR rats were regularly tested with polymorphic markers to confirm their inbred status. At the age of 10 weeks, SHR rats were randomly divided into two groups (SHR group, SHR + HS group), while WKY rats were also randomly divided into two groups (WKY group, WKY + HS group). WKY group and SHR group received a normal-NaCl (0.4%) diet for 10 weeks, whereas WKY + HS group and SHR + HS group received a high-NaCl (4%) diet for 10 weeks.

The article "Hsp90β is involved in the development of high salt-diet-induced nephropathy via interaction with various signalling proteins" was retracted in 2021. Reasons: manipulated images; duplicated images; original data or images not available.

### 2.3. Histological analysis

Paraffin-embedded kidney tissues were cut into sections 4 µm thick. Sections were stained with haematoxylin–eosin (HE) according to conventional histological examination techniques. Analysis of tubules included the evaluation of epithelial histology. The degree of injury was scored semi-quantitatively on a 0–4 scale for reabsorption granules, vacuolization and epithelial degeneration as follows: 0, no lesion; 1, minimal (minor focal changes); 2, mild; 3, moderate; 4, severe. Semi-quantitative analysis of glomeruli included glomerular histology as well as foot process morphology assessed by electron microscopy, and was graded as follows: 1, minimal (involving less than 5% of glomerulus); 2, mild (5–24%); 3, moderate (25–49%); 4, severe (greater than or equal to 50%). Assessment of glomerular involvement, an average of 80–120 glomeruli per section was examined on multiple levels. All scoring was achieved in a blinded manner by an experienced renal pathologist. Semi-quantitative analysis of tubular morphology in rats was also performed in a blinded fashion exactly as described previously [15].

### 2.4. RT-PCR analysis

Total RNA was extracted with Trizol reagent (Gibco) as described by the manufacturer. RT-PCR was performed using the Access RT-PCR Introductory System (Promega) with indicated primers (electronic supplementary material, table S1). PCR was performed for 30 cycles in 25 µl of reaction mixture. PCR products were monitored by microchip electrophoresis system (MultiNA, Shimadzu Biotech, Kyoto). GAPDH was used as a housekeeping gene here.

### 2.5. Treatment of animal models with 17-DMAG

At this stage, 10-week-old SHR rats (*n* = 60) received a high-NaCl (4%) diet for six weeks. SHR rats were also regularly tested with polymorphic markers to confirm their inbred status. Then, these SHR rats were randomly divided into three groups (SHR + HS group, SHR + HS + 0.5 mg kg^−1^ 17-DMAG group and SHR + HS + 2 mg kg^−1^ 17-DMAG group). 17-DMAG was diluted in saline, and its dose was adopted according to previous papers [16]. Rats received 1 ml i.p. administration of 17-DMAG or vehicle (saline) every 2 days for four weeks (from the 16th week to 20th week).

### 2.6. Construction of Hsp90β knockdown cells

The rat cell line, NRK-52E (ATCC, CRL-1571™), was cultured in Dulbecco's modified Eagle's medium (DMEM; Hyclone, Herndon, VA), supplemented with 10% fetal bovine serum (FBS; Gibco, NY) and 1% penicillin and streptomycin (Gibco; Grand Island, NY), and incubated at 5% CO_2_ and 95% humidified atmosphere air at 37°C. The culture medium was replaced twice a week. Once the cells reached confluency, they were passaged using trypsin (0.05%)–EDTA (0.02%) solution. The two recombinant lentiviral expression vectors used in this study were synthesized by Bioworld. One vector expressed Hsp90β-specific siRNA (sense strand: 5′-GAGCTGATACCTGAGTACCTCAACT-3′) and GFP, whereas the other expressed Control siRNA (sense strand: 5′-GCAACCAGGACACTCGTTACATGTT-3′) and GFP. Cells were plated at a density of 2 × 10^5^ cells well^−1^ in six-well culture plates for lentiviral infection. After 24 h, the medium was removed and 1.0 ml DMEM containing 10% FBS, 10 µl (5 × 10^7^) lentivirus and 1 µl (10 mg ml) polybrene (Bioworld, Nanjing) was added to each culture well and gently mixed. After 12 h, the cell culture medium was removed again, and 2 ml DMEM containing 10% FBS and antibiotics was added. Infection was confirmed after 72 h by fluorescence microscopy and little to no toxicity was seen. The cells were passaged and immediately assessed by RT-PCR to ensure the effects of Hsp90β knockdown. Cadmium was added to the medium to induce Hsp90 expression, which could upregulate Hsp90 level in NRK-52E cell line [17].

The article "Hsp90β is involved in the development of high salt-diet-induced nephropathy via interaction with various signalling proteins" was retracted in 2021. Reasons: manipulated images; duplicated images; original data or images not available.

### 2.7. Treatment of animal models with Hsp90β knockdown

At this stage, 10-week-old SHR rats (*n* = 60) received a high-NaCl (4%) diet for six weeks. SHR rats were also regularly tested with polymorphic markers to confirm their inbred status. Then, these SHR rats were randomly divided into three groups (SHR + HS group, SHR + HS + Control siRNA group and SHR + HS + Hsp90β siRNA group). NRK-52E transfectants (1 × 10^6^ cells) expressing either Control siRNA sequence or Hsp90β siRNA sequence were injected into kidneys of SHR + HS rats via the renal artery as previously described [18]. Rats received 1 ml renal arterial injection of vehicle (saline) as control.

### 2.8. Immunoprecipitation and immunoblotting

Tissue samples of whole kidneys were homogenized in ice-cold PBS buffer containing protease inhibitor cocktail, and the total proteins were extracted using NE-PER nuclear and cytoplasmic extraction reagents (Pierce, Rockford, IL), according to the manufacturer's protocol. The protein concentration of tissue supernatant was determined by BioSpec-nano (Shimadzu Biotech, Kyoto). Proteins were immunoprecipitated with indicated antibodies respectively. The precleared Protein A/G Plus–agarose beads (Santa Cruz Biotechnology) were incubated with immunocomplexes for 2 h and washed four times with the lysis buffer. The immunoprecipitates were subjected to SDS–PAGE followed by transferring onto nitrocellulose membranes (Hybond-C, Amersham Biosciences). The immunoblot analysis was performed as described previously [19]. The antibody–antigen complexes were visualized by the LI-COR Odyssey Infrared Imaging System according to the manufacturer's instruction using IRDye800 fluorophore-conjugated antibody (LI-COR Biosciences, Lincoln, NE) or using TMB immunoblotting system (Promega, Madison, WI). Quantification was directly performed on the blot using the LI-COR Odyssey analysis software.

The article "Hsp90β is involved in the development of high salt-diet-induced nephropathy via interaction with various signalling proteins" was retracted in 2021. Reasons: manipulated images; duplicated images; original data or images not available.

### 2.9. Statistics

Data are expressed as mean ± s.e. Statistical analyses were performed by unpaired *t*-test, ANOVA and subsequent Tukey's test or Kruskal–Wallis test followed by Mann–Whitney *U*-test. *p* < 0.05 was considered significant.

## 3. Results

### 3.1. Effects of high-salt diet on blood pressure and proteinuria

We first examined whether a high-salt diet affected blood pressure and proteinuria in WKY/SHR rats. Even at the age of 20 weeks, the SBP of high-salt-diet groups was not considerably higher than the normal-salt-diet group (electronic supplementary material, figure S1). However, the relativity of the relationship between natriuresis and blood pressure tended to be somewhat significant with increasing age, thereby indicating that blood pressure might be sensitive to salt loading with old age. Urinary microalbumin and β2-microglobulin are common nephropathic indicators that reflect the severity of renal pathogenesis. Strikingly, the differences of microalbumin and β2-microglobulin were much more pronounced (electronic supplementary material, figure S1). At the age of 20 weeks, the degree of proteinuria in WKY + HS group was nearly twice that seen in WKY group, and the degree of proteinuria in SHR + HS group even reached three times that of SHR group. Thus, the data implied that non-pressure-related effects of salt loading mainly contributed to its impact on nephropathic outcome.

### 3.2. Effects of high-salt diet on renal histology

HE staining and injury indices showed that high-salt diet indeed caused nephropathy in WKY/SHR rats (figure 1), where renal tubular hyalinecasts enlargement and atrophy were obviously seen in high-salt-diet groups. Meanwhile, hypertension-induced renal arteriole wall thickening was also markedly seen in either SHR group or SHR + HS group. In human renal disease, the reduction in glomerular filtration rate is significantly related to the histological changes observed in the tubules and interstitium. The excess filtered protein reabsorption by the proximal tubules is degraded by lysosomes. When the intracellular products of this degradation reach the interstitial space, they give rise to focal infiltrates of inflammatory cells with an increased deposition of collagen, matrix and fibrous tissue. Our data also yielded that high-salt diet resulted in the inflammatory infiltration and fibrosis of rat kidneys. Moreover, transmission electron microscopy (TEM) analysis revealed severe renal damage, such as renal tubular epithelial cell vacuolization in high-salt-diet groups (electronic supplementary material, figure S2). Interestingly, renal tubular atrophy and epithelial cell vacuolization were usually indicative of epithelial cells undergoing programmed cell death.

The article "Hsp90β is involved in the development of high salt-diet-induced nephropathy via interaction with various signalling proteins" was retracted in 2021. Reasons: manipulated images; duplicated images; original data or images not available.

**Figure 1.** Histological analysis of rat kidney. (*a*) HE staining of WKY group; (*b*) HE staining of WKY + HS group; (*c*) HE staining of SHR group; (*d*) HE staining of SHR + HS group. 1, renal tubular atrophy; 2, renal tubular hyalinecasts; 3, renal tubular enlargement; 4, glomerular fibrosis. (*e*) Injury indices of rat kidney in four groups (*n* = 10 per group; open triangles: statistically significant compared with WKY group; filled triangles: statistically significant compared with SHR group).

### 3.3. Urinary quantitative proteome analysis

Many changes and alterations in kidney functions can be monitored in rat models through urinary proteomic analysis. Here, we performed urine quantitative proteome analysis in either normotensive or hypertensive rats that could specifically reflect non-pressure-related proteomic changes upon salt-loading. Contrasted with WKY group, there were 28 upregulated proteins and 12 downregulated proteins in WKY + HS group (electronic supplementary material, table S2). Moreover, contrasted with SHR group, there were 39 upregulated proteins and 18 downregulated proteins in SHR + HS group (electronic supplementary material, table S3). Among these differentially expressed proteins, 25 upregulated proteins and 10 downregulated proteins were common in WKY + HS group and SHR + HS group (bold in electronic supplementary material, table S2 and S3). Elevated level of fibronectin is usually involved in tissue fibrosis, which can be directly regulated by HIF-1α transcriptionally [20]. Superoxide dismutase [Cu–Zn] was also upregulated, which was involved in excessive renal oxidative stress [21]. On the other hand, EGF, u-PA and cadherin-1 were downregulated in high-salt-diet groups, which were proven to have cytoprotective effects in the kidney, such as the prevention of fibrosis and degradation of accumulated extracellular matrix [22,23]. We finally selected heat shock protein β (Hsp90β) owning to two factors: it was previously proven to regulate the upstream mediators in multiple cellular signalling cascades through stabilizing and maintaining their activities, and it is the only protein possibly involving renal fibrosis, inflammation and tubular epithelial cell death here; it has been rarely seen in previous investigations of salt-loading-induced renal dysfunction.

The article "Hsp90β is involved in the development of high salt-diet-induced nephropathy via interaction with various signalling proteins" was retracted in 2021. Reasons: manipulated images; duplicated images; original data or images not available.

### 3.4. Effects of high-salt diet on nephropathic markers and various cellular signalling pathways

Immunohistochemical analysis of Hsp90β were performed here, and revealed that its expression was indeed elevated in high salt diet groups (electronic supplementary material, figure S3), which was also confirmed by RT-PCR measurements. Interestingly, high-salt diet did not affect Hsp90α expression (figure 2). TGF-β, HIF-1α, TNF-α, IL-6 and MCP-1 expressions were similarly elevated in high-salt-diet groups markedly (figure 2). These nephropathic markers are universal proinflammatory or profibrotic cytokines, which can be directly or indirectly regulated by diverse cellular signalling cascades, such as nuclear factor-kappa B (NF-κB), and mitogen-activated protein kinases (MAPKs) [24]. Therefore, we examined the effects of high-salt diet on NF-κB, extracellular regulated protein kinase (ERK), c-Jun N-terminal kinase (JNK) and p38 MAPK signalling cascades here. The results showed that high-salt diet augmented the activations of NF-κB and p38 MAPK without altering the activations of ERK1/2 and JNK1/2 in high-salt-diet groups (figure 3). Meanwhile, NF-κB nuclear translocation was also increased markedly by high-salt diet (electronic supplementary material, figure S4). In addition, due to the fact that tubular epithelial cell death occurred in high-salt-diet-induced nephropathy, we also examined the effects of salt-loading on Bcl-2 (B-cell lymphoma-2, an anti-apoptotic protein) activation, and the data showed that it indeed led to the phosphorylation/inactivation of Bcl-2.

**Figure 2.** RT-PCR analyses of high-salt-diet-induced renal Hsp90β, TGF-β, HIF-1α, TNF-α, IL-6, MCP-1 and Hsp90α expression (*n* = 5 per group; open triangles: statistically significant compared with WKY group; filled triangles: statistically significant compared with SHR group; GAPDH as internal standard).

**Figure 3.** Measurement of high-salt-diet-mediated ERK1/2, JNK, p38 and NF-κB activation and Bcl-2 inactivation in rat kidney. Renal Phospho-ERK1/2, ERK1/2, phospho-JNK1/2, JNK1/2, phospho-p38, p38, phospho-Bcl-2, Bcl-2, phospho-IκBα and IκBα expressions were detected by Western blot assay (*n* = 5 per group; open triangles: statistically significant compared with WKY group; filled triangles: statistically significant compared with SHR group; β-actin as internal standard).

The article "Hsp90β is involved in the development of high salt-diet-induced nephropathy via interaction with various signalling proteins" was retracted in 2021. Reasons: manipulated images; duplicated images; original data or images not available.

### 3.5. Effects of Hsp90β inhibition on blood pressure, proteinuria and renal histology

In this study, SHR rats developed more severe nephropathy than WKY rats in response to high-salt diet, because essential hypertension is often characterized to induce vascular remodelling (VR). VR mainly involves thickening of the arterial wall, and this change also facilitates the development of tissue damage [25]. Thus, we selected SHR + HS group as the target of Hsp90β inhibition in this study. A water-soluble Hsp90 inhibitor, 17-DMAG, was administrated to investigate the role of Hsp90β in high-salt-diet-induced nephropathy. On the other hand, Hsp90β siRNA was also transfected into rat kidneys to improve the specificity of Hsp90β inhibition, whereas immunohistochemical analysis confirmed the effects of Hsp90β knockdown *in vivo* (electronic supplementary material, figure S5). It was demonstrated that Hsp90β inhibition hardly affected the SBP of SHR + HS group (electronic supplementary material, figure S6*a*,*d*). However, urinary secretion of microalbumin and β2-microglobulin was reversed significantly by 17-DMAG dose-dependently (electronic supplementary material, figure S6*b*,*c*), and this effect was also confirmed by treatment with Hsp90β knockdown (electronic supplementary material, figure S6*e*,*f*). HE staining and TEM analysis were carried out to evaluate the effects of Hsp90β inhibition on renal histology. We discovered that 17-DMAG or Hsp90β knockdown significantly impaired glomerular fibrosis, renal tubular hyalinecasts, enlargement and atrophy (figure 4), and renal tubular epithelial cell vacuolization was also relieved by Hsp90β inhibition (electronic supplementary material, figure S7).

**Figure 4.** Histological analysis of rat kidney treated with 17-DMAG or Hsp90β knockdown. (*a*) HE staining of SHR + HS group (rats received i.p. administration of saline); (*b*) HE staining of SHR + HS + 0.5 mg kg^−1^ 17-DMAG group; (*c*) HE staining of SHR + HS + 2 mg kg^−1^ 17-DMAG group; (*d*) injury indices of rat kidney in (*a*), (*b*) and (*c*) groups; (*e*) HE staining of SHR + HS group (rats received renal arterial injection of saline); (*f*) HE staining of SHR + HS + Control siRNA group; (*g*) HE staining of SHR + HS + Hsp90β siRNA group; H injury indices of rat kidney in (*e*), (*f*) and (*g*) groups (*n* = 10 per group; open triangles: statistically significant compared with SHR + HS group).

### 3.6. Effects of Hsp90β inhibition on nephropathic markers and related cellular signalling pathways

Contrasted with SHR + HS group, 17-DMAG or Hsp90β knockdown reversed the phosphorylations of inhibitor of NF-κB α (IκBα), Bcl-2 and p38 MAPK, without altering their protein expressions (figure 5). Meanwhile, NF-κB nuclear translocation was impaired significantly by Hsp90β inhibition (electronic supplementary material, figure S8). Next, we examined the effects of Hsp90β inhibition on upstream kinases of NF-κB and p38, including mitogen-activated protein kinase kinase 3 (MKK3/6) and IKKα/β (IκB kinase α/β). The results showed that 17-DMAG or Hsp90β knockdown also reversed the phosphorylation of IKKα/β in SHR + HS rats, suggesting that Hsp90β is required for the protein stability of IKK. Surprisingly, MKK3/6 activation was not affected by Hsp90β inhibition. It was suspected that p38 activation might be regulated via other uncanonical activators. MKK3/6-independent p38 activation is usually associated with TAK1-binding protein 1 (TAB-1) interaction, when active AMP-activated protein kinase (AMPK) can trigger p38 recruitment to TAB1 and p38 autophosphorylation [26,27]. Our data revealed that Hsp90β inhibition reversed TAB-1-mediated p38 phosphorylation via inactivation of AMPKα (electronic supplementary material, figure S9). In addition, mammalian target of rapamycin (mTOR) phosphorylates and activates ribosomal protein S6 kinase (p70S6 K, Thr389), which is also involved in the phosphorylation/inactivation of Bcl-2. Inactivation of Bcl-2 triggers the release of cytochrome *c* from mitochondria, leading to the activations of downstream pro-apoptotic caspases [28]. Our data also showed that 17-DMAG or Hsp90β knockdown indeed reversed the activations of mTOR/p70S6 K and the release of cytochrome *c* (figure 6), suggesting that Hsp90β promotes the tubular epithelial cell apoptosis mediated by mTOR signalling.

The article "Hsp90β is involved in the development of high salt-diet-induced nephropathy via interaction with various signalling proteins" was retracted in 2021. Reasons: manipulated images; duplicated images; original data or images not available.

**Figure 5.** Hsp90β inhibition reversed various signalling cascades of rat kidney treated with 17-DMAG or Hsp90β knockdown. Renal phospho-IKKα/β, IKKα/β, phospho-IκBα, IκBα, phospho-MKK3/6, MKK3/6, phospho-AMPKα, AMPKα, phospho-p38, p38, phospho-Bcl-2 and Bcl-2 expressions were detected by Western blot assay. (*a*) 17-DMAG reversed various signalling cascades of rat kidney in SHR + HS group that received i.p. administration of saline; (*b*) Hsp90β knockdown reversed various signalling cascades of rat kidney that received renal arterial injection of saline (*n* = 5 per group; open triangles: statistically significant compared with SHR + HS group; β-actin as internal standard).

**Figure 6.** Hsp90β inhibition reversed tubular epithelial cell apoptosis of rat kidney treated with 17-DMAG or Hsp90β knockdown. (*a*) 17-DMAG reversed phospho-mTOR, phospho-p70S6 K and cytochrome *c* expressions of rat kidney in SHR + HS group that received i.p. administration of saline; (*b*) Hsp90β knockdown reversed phospho-mTOR, phospho-p70S6 K and cytochrome *c* expressions of rat kidney that received renal arterial injection of saline (*n* = 5 per group; open triangles: statistically significant compared with SHR + HS group; β-actin as internal standard).

### 3.7. Effects of Hsp90β inhibition on endogenous Hsp90β protein complex and renal oxidative stress

A variety of signalling proteins involved in cell survival, growth and differentiation are recognized as Hsp90 client proteins. On ATP binding, the Hsp90 client complex associates with co-chaperones such as cell division cycle 37 (CDC37) and p23 to facilitate client stabilization. Here, we investigated whether Hsp90β inhibition affected the stability of some potential Hsp90β client proteins in rat kidneys (figure 7). The results demonstrated that 17-DMAG or Hsp90β knockdown effectively reduced the interactions of TAK1 (TGF-β-Activated Kinase 1), AMPKα, IKKα/β, HIF-1α and Raptor (regulatory-associated protein of TOR, an important positive regulatory subunit of mTOR complex) with Hsp90β, indicating that endogenous Hsp90β protein complex was required to maintain the high-salt-diet-induced nephropathy. In addition, we measured the urinary secretion of 8-OHdG (8-hydroxy-2′-deoxyguanosine, an indicator of renal oxidative stress; electronic supplementary material, figure S10). Compared with normal-salt-diet groups, high-salt-diet induced greater renal oxidative damage. However, 17-DMAG or Hsp90β knockdown decreased the urinary secretion of 8-OHdG in SHR + HS group. In spite of the effects of Hsp90β on ROS-mediated cellular signalling pathways, our results indicated that Hsp90β was also required for excessive renal oxidative stress in salt-loaded rats.

**Figure 7.** Hsp90β inhibition disrupted the Hsp90β protein complex of rat kidney, including: (*a*) 17-DMAG disrupted the Hsp90β protein complex of rat kidney in SHR + HS group that received i.p. administration of saline; (*b*) Hsp90β knockdown disrupted the Hsp90β protein complex of rat kidney in SHR + HS group that received renal arterial injection of saline. Hsp90β, TAK1, AMPKα, IKKα/β, HIF-1α and Raptor expressions were detected in either Hsp90β protein complex or total cell lysates of rat kidney (rIgG as rabbit control IgG, β-actin as internal standard).

## 4. Discussion

Here, we identified a novel mechanism of high-salt-diet-induced nephropathy, including renal inflammation, fibrosis and tubular epithelial cell apoptosis. Our data showed for the first time that, to the best of our knowledge, high-salt-diet-induced nephropathy was specifically associated with enhanced levels of Hsp90β, which played the key role in non-pressure-related effects of salt loading. However, Hsp90α, another important isoform of Hsp90, tended to be sensitive to hypertension instead of salt loading in this study. It indicated that Hsp90α and Hsp90β might exhibit significantly different behaviours under stress conditions, though they had similar interactions with co-chaperones.

The article "Hsp90β is involved in the development of high salt-diet-induced nephropathy via interaction with various signalling proteins" was retracted in 2021. Reasons: manipulated images; duplicated images; original data or images not available.

The majority of renal oxygen consumption results from reabsorption of approximately 99.5% of filtered sodium, so the increased kidney metabolism is usually associated with high-salt diet, as well as the decreased renal oxygen availability in both animals and patients. This change directly results in renal hypoxia, which often leads to the overexpression of HIF-1. Here, HIF-1 was indeed increased dramatically in response to salt loading in WKY/SHR. HIF-1 is often responsible for renal fibrosis. Here, our *in vivo* data showed that Hsp90β protected HIF-1α in high-salt-diet-induced nephropathy, which was reversed by 17-DMAG or Hsp90β knockdown. Hsp90 has been reported to induce the stabilization of HIF-1α [29]. Thus, Hsp90β inhibition resulted in the decreased expression of HIF-1α, leading to the impaired transcriptional regulatory activity of HIF-1. In this study, the expression of TGF-β (a key downstream target gene of HIF-1) was indeed reduced by Hsp90β inhibition, and the TGF-β-mediated renal fibrosis obtained effective restriction simultaneously.

In the kidney, a high salt intake often favours not only renal hypoxia, but also renal oxidative stress. The reason might be that hypoxia could accumulate ROS in renal tissue, and this oxidative stress conversely facilitated renal hypoxia owing to inefficient cellular respiration. *In vitro* COS-7 cell experiments previously demonstrated that Hsp90 could interact with Nox5, and was required for enzyme stability and ROS production of Nox [30]. Our *in vivo* data also yielded that secretion of urinary 8-OHdG was strikingly elevated in response to salt loading, and reversed by Hsp90β inhibition.

Besides the direct effect on renal oxidative stress, Hsp90β might also affect ROS-mediated renal inflammation and tubular epithelial cell apoptosis together. Pro-inflammatory cytokines, such as TNF-α, IL-6 and MCP-1, were indeed induced substantially in response to salt loading, which could be transcriptionally regulated by NF-κB or p38 MAPK signalling cascades. Our results showed that high-salt diet simultaneously promoted the inflammatory response via NF-κB and p38 MAPK activations in rat kidneys, which were markedly reversed by 17-DMAG or Hsp90β knockdown. Here, Hsp90β maintained the protein stability of IKK, and IKK activated downstream IκBα, where inactivated IκBα blocked the transcriptional regulatory activity of NF-κB. Decreased nuclear translocation of NF-κB confirmed the role of Hsp90β inhibition. Similarly, Hsp90β inhibition might induce the degradation of AMPKα, and cause a significant decrease in enzyme ability of AMPKα, where AMPKα–TAB1 complex maintained the kinase activity of p38. More importantly, Hsp90β inhibition significantly suppressed salt-loading-stimulated expression of TAK1, where TAK1–TAB1 complex maintained the kinase activity of IKK. In addition, HIF-1α has been reported to be phosphorylated by p38 directly, and NF-κB could stimulate the transcription of HIF-1α gene [31,32]. Thus, there might be a cross-talk between renal inflammation and fibrosis.

The article "Hsp90β is involved in the development of high salt-diet-induced nephropathy via interaction with various signalling proteins" was retracted in 2021. Reasons: manipulated images; duplicated images; original data or images not available.

On the other hand, high-salt-diet-induced oxidative stress damages epithelial cells directly, causing the tubular epithelial cell death. mTOR may have a pleiotropic function in the regulation of cell apoptosis [28]. The binding of raptor to mTOR is required for the mTOR-catalysed phosphorylation of downstream effectors, where it strongly enhances the mTOR kinase activity towards p70S6 K [33]. Activation of mTOR and downstream target p70S6 K is associated with increased inactivation of Bcl-2 and release of cytochrome *c* from mitochondria to cytoplasm, suggesting that the mTOR pathway plays a critical role in the apoptosis of renal tubular epithelial cells in response to salt loading. Our results showed that 17-DMAG or Hsp90β knockdown impaired the protein stability of Raptor, and this change resulted in the suppression of mTOR activity. Thus, Hsp90β inhibition might relieve the renal tubular epithelial cell apoptosis via downregulating mTOR-p70S6 K-Bcl2 axis, and the reduction of renal tubular epithelial cell vacuolization confirmed this point. Moreover, IKK has been reported to phosphorylate and inactivate tuberous sclerosis protein 1, which could facilitate the activation of mTOR signalling [34]. It indicated that renal inflammation might not only promote renal fibrosis reciprocally, but also affect the renal tubular epithelial cell apoptosis. In this study, the reduction of pro-inflammatory cytokines by Hsp90β inhibition indeed accompanied the downregulation of HIF-1-mediated fibrosis and Bcl-2-mediated cell death.

As a conclusion, the renal hypoxia and oxidative stress driven by high-salt diet promoted the progress of renal damage, including renal inflammation, fibrosis and tubular epithelial cell apoptosis. Hsp90β maintained the stability and activity of various cellular signalling proteins, which might be required for non-pressure-related effects of high-salt-diet-induced nephropathy (figure 8). We also believed that the regulatory functions of Hsp90β would not be merely confined to our study, because the latest discovery revealed that 17-DMAG also ameliorated diabetic nephropathy via the suppression of NF-κB and STAT (signal transducers and activators of transcription) signalling in experimental mice [35]. All these factors suggest that Hsp90β has potential therapeutic value in high-salt-diet-induced nephropathy.

The article "Hsp90β is involved in the development of high salt-diet-induced nephropathy via interaction with various signalling proteins" was retracted in 2021. Reasons: manipulated images; duplicated images; original data or images not available.

**Figure 8.** Hsp90β stabilized TAK1, then TAK1 activated IKKα/β, then IKKα/β promoted the ubiquitination of IκBα, leading to the subsequent NF-κB signalling; Hsp90β interacted with HIF-1α, and maintained its activity; Hsp90β directly stabilized IKKα/β, leading to the subsequent NF-κB signalling; Hsp90β stabilized AMPKα, then AMPKα induced the TAB1-mediated p38 activation; Hsp90β stabilized Raptor, resulting in mTOR-mediated tubular epithelial cell apoptosis. All these cellular effects resulted in renal fibrosis, inflammation and apoptosis.
